The article "Research on Image Feature Extraction Algorithm of the Egg and Egg White Protein Thermal Gelation Based on PCA/ICA" was published in 2022. Journal: Comput Intell Neurosci.

# Research on Image Feature Extraction Algorithm of the Egg and Egg White Protein Thermal Gelation Based on PCA/ICA

**DOI:** 10.1155/2022/1266332

**Published:** 2022-03-26

**Authors:** XinCi Liu, Chang Zhao

**Affiliations:** ^1^School of Food Engineering, Harbin University of Commerce, Harbin 150028, China; ^2^School of Food Engineering, Heilongjiang Vocational College for Nationalities, Harbin 150066, China

## Abstract

With the rapid development of the computer field in recent years, a series of major breakthroughs have been made in the field of computer vision. The key technologies in image feature recognition, face recognition, image understanding, pattern recognition, and machine learning have been rapidly applied and developed. The research and application of this field provide efficient and convenient means. However, for traditional physical and chemical experimental research, parameter adjustment is time-consuming and costly. In response to the phenomenon, this article starts with the study of the characteristics of the egg white protein thermal gelation image and explores the extraction of external features presented by the optimal parameters of the coagulation image under the thermal coagulation state of the egg white protein, based on the classic PCA and ICA—image feature extraction algorithm and its improved algorithm, respectively. Experiment and simulation research on several image feature extraction algorithms under different egg white solidification states are carried out, and the efficient recognition method and accuracy of the image under the optimal egg white protein thermal gelation state are discussed. It has important reference significance for the research of optimal image feature extraction in the future high-efficiency experimental research.

## 1. Introduction

Image feature extraction is a process of extracting multiple unique attributes from the preprocessed image target, so that the extracted features reflect the characteristics of the image target as much as possible. This technology is the basis for image object classification, recognition, tracking, and other computer vision-related applications. It is a key link in the image processing process, as well as a key technology for image understanding, pattern recognition, and machine learning. In the image feature extraction, the gray-scale feature of the image pixel and the statistical feature of the pixel's gray-scale value are the most easily obtained features. Extracting images of the best physical and chemical experimental state, avoiding the need to coordinate various parameters in the past, and finding the best state to spend a lot of time and manpower cost have important reference significance. The optimal state image is often produced in physics and chemistry research, and the optimal solution of each parameter is determined by the characteristics of the algorithm. In recent years, with the rapid development of the computer field, a series of major breakthroughs have been made in the field of computer vision, providing efficient and convenient means for research and application in various fields. This thesis starts with the image feature research of the egg white protein thermal gel. Based on the classic PCA and ICA image feature extraction algorithms, as well as several existing improved algorithms, experimental simulation studies are carried out on these image feature extraction algorithms.

The article "Research on Image Feature Extraction Algorithm of the Egg and Egg White Protein Thermal Gelation Based on PCA/ICA" was published in 2022. Journal: Comput Intell Neurosci.

## 2. Related Work

Feature extraction is one of the most fundamental problems in the field of pattern recognition. Extracting effective discrimination features is a prerequisite for solving the problem of target classification and recognition. The research of feature extraction mainly has the following two purposes: one is to find the most discriminative description between targets, so that different types of targets can be separated from each other; and the other is to compress the dimensionality of target data under certain circumstances.

According to whether it can be linearly separable, the feature extraction methods can be divided into two types: one is the linear feature extraction method, and the other is the nonlinear feature extraction method [1]. To date, for the problem of linear separable feature extraction, people have given many solutions, including principal component analysis [2, 3] (PCA), independent component analysis [4] (ICA), factor analysis (FA), locality preserving projections [5] (LPP), linear discriminant analysis [6] (LDA), local feature analysis (LFA), multidimensional scaling (MDS) is the most classic and widely used method in linear feature extraction algorithms. The linear feature extraction method is easy to understand and easy to implement. It has been successfully applied to various problems such as face recognition, character recognition, speech recognition, and text classification. Aiming at the problem of complex nonlinear separable feature extraction, the introduction of nuclear technology has become one of the important methods to solve. The core idea is to project in a low-dimensional space so that it is linearly separable and then use linear methods for processing.

Principal component analysis is a classic feature extraction algorithm. As early as 1873, Beltrami and Jordan independently derived PCA on the basis of singular value decomposition (SVD). In 1933, the geometric description and algebraic description of PCA were given. In 1967, Jeffers used PCA in practical situations and not just as a dimensionality reduction tool. Jian Yang et al. proposed two-dimensional principal element analysis in 2004 [7–10] (two-dimensional principle component analysis—2DPCA). There is no need to convert a two-dimensional image matrix into one-dimensional data, so it does not change the neighboring relationship of image pixels, which can more accurately estimate the covariance matrix of the image. In recent years, with the widespread application of tensors, Haiping Lu et al. proposed multilinear principal component analysis [2, 11, 12] (MPCA), which extended PCA from one-dimensional vector space to multidimensional tensor space.

The article "Research on Image Feature Extraction Algorithm of the Egg and Egg White Protein Thermal Gelation Based on PCA/ICA" was published in 2022. Journal: Comput Intell Neurosci.

Independent component analysis, as an extension of PCA, focuses on the high-order statistics between the data, so that the high-order statistics between the transformed components are independent, and can reflect the essential characteristics of the data. In 2006, Hyvarinen proposed Fast ISA, a fast algorithm for ISA, which has good convergence and reduces the running time of the algorithm. In 2009, Hyvarinen used ISA in the feature extraction and analysis of natural images, which well reflected the essential characteristics of natural images. Scholars at home and abroad [13–18] have developed rapidly in the past 10 years on the algorithm and application of ICA, such as the Computational Neurobiology Laboratory of the Department of Biology, University of California, the Computer and Information Science Laboratory of Helsinki University of Technology in Finland, the Riken Institute of Brain Science in Japan, and the Intelligent Perception and Image Understanding of the Ministry of Education in Xidian University.

The task of image feature extraction is to map data samples in a high-dimensional space to a low-dimensional feature space, so that the statistical correlation between the extracted features is as small as possible, and the separability between different types of features is a certain classification, which is best maintained or enhanced in advance. Principal component analysis considers that the image has a Gaussian distribution, focuses on the two-dimensional statistics of the image, and decorrelates the image. Independent component analysis not only involves the second-order correlation between the images, but also relates to the high-order independence—which is an extension of PCA. The previous research on white protein in egg mainly stayed on the microscopic study of characteristics, and these lacked the study of characteristics to reflect the changes of its parameters. This article will use PCA and ICA to enhance the advantages of the distinguishing ability of characteristics to varying degrees. Corresponding research is also an important development direction for future research on microfeature parameter extraction. This article will use PCA and ICA to enhance the advantages of the distinguishing ability of characteristics to varying degrees. Corresponding research is also an important development direction for future research on micro-feature parameter extraction.

The article "Research on Image Feature Extraction Algorithm of the Egg and Egg White Protein Thermal Gelation Based on PCA/ICA" was published in 2022. Journal: Comput Intell Neurosci.

## 3. Image Feature Analysis of Thermal Gelation of the Egg White Protein

### 3.1. Experimental Method

#### 3.1.1. Egg White Preparation

First, the egg whites of fresh eggs were separated manually, then stirred with a high-speed disperser (speed 35r/s) for 20 minutes, allowed them stand for 1 hour to discard the bottom umbilical cord and other impurities, and finally placed in a refrigerator at 4 °C for later use.

#### 3.1.2. Moisture Content Determination

Moisture content was determined by oven-drying method.

#### 3.1.3. Preparation of Gel and Determination of Gel Strength

The egg white was diluted with distilled water to the set concentration. According to GB 2760–2007 Food Additives Hygiene Standard, after the addition of food additives or ingredients below the allowable amount to the above diluted egg white, 35 mL was taken into a 50-mL beaker, sealed with plastic wrap, and used after heating in a water bath for a certain period of time. It is cooled in an ice-water bath, placed in a refrigerator at 4 °C for 14 hours, and then taken out for use (Christ Det al., 2005).

The coagulation strength of the egg white expressed was tested by P0.5 probe of the physical property tester with the measured hardness, parallel sample (n = 6) (Valerie Lechevalier et al. 2007 ). The measurement conditions are as follows:

  Speed before test: 5 mm/s;
  Testing speed: 1 mm/s;
  Speed after measurement: 5 mm/s;
   Compression ratio: 50%;
  Trigger force: 5g.

#### 3.1.4. Differential Scanning Calorimetry

Netzsch DSC 204 F1 differential scanning calorimetry (DSC) was used to study the thermal characteristics of the egg whites. Pure metal indium (99.99%) was used to correct the enthalpy and temperature of the instrument. 20 mg of egg white sample was weighed with a solid content of 10% into a 25 *μ*l aluminum crucible. Then, the sample is sealed and the distilled water of the corresponding quality is used as a reference. The temperature is increased from 30 °C to 100 °C at a heating rate of 2 °C·min^−1^. The whole process is carried out under dry N2, the flow rate of purge gas is 20 ml·min^−1^, and the flow rate of shielding gas is 60 ml·min^−1^ (Yoshinori Mine, 1996).

### 3.2. Image Feature Analysis of Thermal Gelation of the Egg White Protein

The egg white begins to thicken at 60 °C, but when the gel temperature is lower than 70 °C, the gel strength formed is extremely low. It can be seen from Figure 1 that the gel strength increases with the setting between 80 °C and 90 °C. The temperature of the gel increases; the strength of the gel does not increase at a temperature greater than 90 °C and remains basically stable, but the pores in the gel gradually increase, and a large number of pores are generated at 100 °C, and a relatively stable gel strength value cannot be measured. Considering that it is necessary to obtain a gel with high gel strength and to ensure stable test results, the gel temperature for the following tests is selected as 90 °C.

The article "Research on Image Feature Extraction Algorithm of the Egg and Egg White Protein Thermal Gelation Based on PCA/ICA" was published in 2022. Journal: Comput Intell Neurosci.

It can be seen from Figure 2 that when the gel temperature is 90 °C, when the gel time is less than 30 minutes, the gel strength increases with the increase of the gel time; the fresh egg white and the egg white with a solid content of 10% are all congealing. When the gel time is 30 minutes, the gel solidification transition reaches the maximum; after 30 minutes, the gel solidification transition remains stable and no longer increases with the extension of the gel time, but the gel turns brown when the gel time is greater than 50 minutes. Based on the above research conclusions, for the convenience of image feature research, for the subsequent research on the egg and egg white protein thermal gelation image feature extraction algorithm, the egg white with a solid content of 10%, gel temperature of 90 °C, gel time of 30 min, and image feature recognition are selected. The image features in this state are stable, and the best egg gel state can be judged by direct recognition, which can provide a reference for relevant experimental research with efficient research methods.

## 4. Analysis of Feature Extraction Algorithm of the Egg and Egg White Protein Thermal Gelation Image Based on PCA/ICA

### 4.1. Feature Extraction of Thermal Gelation Image of the Egg and Egg White Protein Based on PCA

#### 4.1.1. PCA

The classic PCA-based image feature extraction algorithm directly performs feature extraction on the pixel gray level of the image, which is easy to understand and easy to implement, but only considering the pixel gray value information cannot meet the feature extraction of complex images. The PCA algorithm is improved through image pre-transformation, one-dimensional to multidimensional, and block sub-models. The structure information of the image is used to greatly reduce the dimension of the image matrix during operation. At the same time, the image is decomposed by wavelet transform and wavelet is used. The coefficient describes the image, which can effectively extract detailed information and reduce the complexity of subsequent calculations. Wavelet PCA [19] first uses wavelet transform to preprocess the image to obtain a wavelet image that is much smaller than the original image dimension, and then uses the PCA algorithm for feature extraction, which can effectively extract the main features of the image and reduce the algorithm complexity.

The article "Research on Image Feature Extraction Algorithm of the Egg and Egg White Protein Thermal Gelation Based on PCA/ICA" was published in 2022. Journal: Comput Intell Neurosci.

The purpose of the PCA algorithm is to find an optimal feature subspace, so that the observation data are projected under this feature subspace, and the component with the largest variance is obtained. It is to find an orthogonal transformation matrix W, so that after orthogonal transformation of the multidimensional data, the new components after transformation are not related to each other.

Suppose *X*=(*x*_1_, *x*_2_,…,*x*_*n*_)^*T*^ is an n-dimensional random variable, and its mean value can be expressed as follows:

(1) $$\begin{array}{c} \bar{x}=\frac{1}{N}\sum_{n-1}^{N}x_{n}. \end{array}$$

After de-averaging *X*, the component obtained by PCA processing can be expressed as *y*_*i*_=*w*_*i*_^*T*^*X*. The feature extraction process of PCA can be described as when the observation data are projected into the feature space, first by looking for *w*_1_, *y*_1_=*w*_1_^*T*^*X* has the largest variance, and *y*_1_ is called the first principal component (PC1). Next, by looking for *w*_2_, *y*_2_=*w*_2_^*T*^*X* has the second largest variance, and *y*_1_ and *y*_2_ are not correlated, and *y*_2_ is called the second principal component (PC2). By analogy, *y*_*k*_=*w*_*k*_^*T*^*X* has the *k*th largest variance and is uncorrelated with the previously determined *y*_1_, *y*_2_,…*y*_*k*−1_. Then *y*_*k*_ is called the *k*th principal component (PC *k*) Until all principal components are found {*y*_*i*_*|i*=1,2,…*n*}.  Figure 3 shows the principal component directions of a set of two-dimensional zero-mean random data, where X_1_ and X_2_ are the original coordinate directions, PC1 and PC2 are the principal component directions after PCA processing, and PC1 and PC2 are not correlated with each other.

In fact, a few principal components can meet the demand for data information, that is, the orthogonal transformation matrix {*w*_*i*_=*i*=1,2,…, *n*}, the subscript *p* ≤ *n* in *w*=(*w*_1_, *w*_2_,…, *w*_*p*_), and the principal component is *Y*=(*y*, *y*_2_,…, *y*_*P*_). PCA outputs a few principal components that are not related to each other, which retains the main information of the data and realizes data compression and second-order redundant data removal.

For general natural data, the covariance matrix *C*=*E*[XX^*T*^] is usually a positive definite matrix, and there must be a singular value decomposition *C*=UVU^*T*^, where *U*=(*u*_1_, *u*_2_,…, *u*_*n*_) is the covariance matrix. An orthogonal matrix composed of eigenvectors, *V*  = diag (*λ*_1_, *λ*_2_,…, *λ*_*n*_), is a diagonal matrix composed of eigenvalues corresponding to the eigenvectors. When the eigenvalue satisfies *λ*_1_ > *λ*_2_ > ⋯>*λ*_*n*_, the basis vector of U constitutes the optimal projection matrix of PCA. After the observation data are projected accordingly, the components are not correlated with each other, and the variance of each component is equal to the corresponding characteristic value. The minimum mean square error of the reconstructed data can be expressed as follows:

(2) $$\begin{array}{c} \varepsilon_{m_{i}n}=\sum_{i-p+1}^{n}\lambda_{i}. \end{array}$$

In the image feature extraction, the image is firstly vectorized, and the image f(x, y) with the size of *m*×*n* is connected end-to-end to form a vector *χ* of mn ×1, as shown in Figure 4.

The article "Research on Image Feature Extraction Algorithm of the Egg and Egg White Protein Thermal Gelation Based on PCA/ICA" was published in 2022. Journal: Comput Intell Neurosci.

Assuming that the image training set has *M* training samples, vectorize them to get: {*χ*_*i*_*|i*=1,2,…, *M*}. Then the average vector of *M* images is as follows:

(3) $$\begin{array}{c} \mu =\frac{1}{M}\sum_{i=1}^{M}\chi_{i}. \end{array}$$

Then the covariance matrix of the training image set can be expressed as follows:

(4) $$\begin{array}{c} C=\frac{1}{M}\sum_{i=1}^{M}\left(\chi_{i}-\mu \right){\left(\chi_{i}-\mu \right)}^{T}\\ =\frac{1}{M}{\text{XX}}^{T}. \end{array}$$

Since the size of XX^*T*^ is *mn* × *mn*, for example, the size of the image in the egg white protein image database is 112×92. The high dimensionality of XX^*T*^ makes the calculation of the eigenvectors of the covariance matrix very complicated, and the size of *X*^*T*^*X* is *M*×*M*, usually the number of samples is less than 1000. Assuming that *λ* and *η* are an eigenvalue of XX^*T*^ and the corresponding eigenvector, there are:

(5) $$\begin{array}{c} X^{T}X\eta =\lambda \eta . \end{array}$$

Multiply both sides of the equation by *X* at the same time to get:

(6) $$\begin{array}{c} \left({\text{XX}}^{T}\right)X\eta =\lambda X\eta . \end{array}$$

It can be seen that when the eigenvalues of XX^*T*^ and *X*^*T*^*XX* are the same, the eigenvector is *Xη*. Therefore, the eigenvalues and eigenvectors of the image covariance matrix are calculated by this method.

The feature vectors are sorted according to the size of the feature value. The feature vector corresponding to the larger the feature value is more able to reflect the image feature, and the size of the feature value decreases exponentially. The image corresponding to the feature vector is called a feature sub-image.  Figure 5 is the six-feature sub-images obtained by PCA of the egg and egg white protein image database in the case of five training samples. From left to right, the feature value gradually becomes smaller. It can be seen that the smaller the feature value, the more blurred the feature description and the less information it contains.

The article "Research on Image Feature Extraction Algorithm of the Egg and Egg White Protein Thermal Gelation Based on PCA/ICA" was published in 2022. Journal: Comput Intell Neurosci.

#### 4.1.2. Wavelet PCA

The classic PCA-based image feature extraction algorithm directly performs feature extraction on the pixel gray level of the image, which is easy to understand and easy to implement, but only considering the pixel gray value information cannot meet the feature extraction of complex images. Using wavelet transform to decompose the image and describing the image with wavelet coefficients can effectively extract detailed information and reduce the complexity of subsequent calculations. Wavelet PCA [19] first uses wavelet transform to preprocess the image to obtain a wavelet image that is much smaller than the original image dimension, and then uses the PCA algorithm for feature extraction, which can effectively extract the main features of the image and reduce the algorithm complexity.

Let *f*(*x*) be the original signal, the continuous wavelet transform can be expressed as

(7) $$\begin{array}{c} \text{CWT}\left(a,\tau \right)=\frac{1}{\sqrt{a}}\int_{-\infty }^{\infty }f\left(x\right)\psi \left(\frac{x-\tau }{a}\right)\text{d}x. \end{array}$$

Among them, *ψ* is the mother wavelet function, *a* is the scale variable, and *τ* is the position variable.

The discrete wavelet transform can be defined as follows:

(8) $$\begin{array}{c} \text{CWT}\left(j,k\right)=\frac{1}{\sqrt{2^{j}}}\int_{-\infty }^{\infty }f\left(x\right)\psi \left(\frac{x}{2}-k\right)\text{d}x. \end{array}$$

Among them, *ψ* is the mother wavelet function, *j* is the scale variable, and *k* is a constant.

The image *f*(*x*, *y*) is two-dimensional data, which needs to be decomposed by two-dimensional discrete wavelet transform. The image after two-dimensional discrete wavelet transform can be expressed as follows:

(9) $$\begin{array}{c} f\left(x,y\right)=\sum_{p\cdot q}c_{p,q}\varphi_{p,q}+\sum_{p\cdot q}d_{p,q}^{1}\psi_{p,q}^{1}+\sum_{p,q}d_{p,q}^{2}\psi_{p,q}^{2}+\sum_{p,q}d_{p,q}^{3}\psi_{p,q}^{3}. \end{array}$$

Among them, *c*_*p*,*q*_, *d*_*p*,*q*_^1^, *d*_*p*,*q*_^2^, and *d*_*p*,*q*_^3^ are two-dimensional discrete wavelet coefficients, and *c*_*p*,*q*_=*f*, *φ*_*p*,*q*_, *d*_*p*,*q*_^1^=*f*, *ψ*_*p*,*q*_^1^, *d*_*p*,*q*_^2^=*f*, *ψ*_*p*,*q*_^2^, and *d*_*p*,*q*_^3^=*f*, *ψ*_*p*,*q*_^3^. *φ*_*p*,*q*_ is the scaling function in the two-dimensional discrete wavelet transform; *p* and *q* are the horizontal and vertical displacement marks of the scaling function, respectively; *φ*_*p*,*q*_(*x*, *y*)=*φ*_*p*_(*x*)*φ*_*q*_(*y*). *ψ*_*p*,*q*_^1^, *ψ*_*p*,*q*_^2^, *ψ*_*p*,*q*_^3^ are two-dimensional wavelet functions, which are as follows:

(10) $$\begin{array}{c} \psi_{p,q}^{1}=\varphi_{p}\left(x\right)\varphi_{q}\left(y\right),\\ \psi_{p,q}^{2}=\varphi_{p}\left(x\right)\varphi_{q}\left(y\right),\\ \psi_{p,q}^{3}=\varphi_{p}\left(x\right)\varphi_{q}\left(y\right). \end{array}$$

Four sub-band images can be obtained after one-layer decomposition of two-dimensional discrete wavelet transform. Among them, the LL sub-band image retains the low-frequency components of the original image, which is also called a smooth image; HL retains the horizontal details of the original image; LH retains the vertical details of the original image; and HH retains the oblique edge details of the original image.  Figure 6 is the result of one-layer wavelet transformation of the egg white thermal gel image in the egg white protein image database using the dB2 wavelet of the Daubechies wavelet series. Usually, we replace the original image with the LL sub-band image after wavelet decomposition for PCA feature extraction. The LL sub-band image is much smaller than the size of the original image matrix, which can effectively improve the real-time performance of the algorithm.

The article "Research on Image Feature Extraction Algorithm of the Egg and Egg White Protein Thermal Gelation Based on PCA/ICA" was published in 2022. Journal: Comput Intell Neurosci.

### 4.2. Feature Extraction of the Egg and Egg White Protein Thermal Gelation Image Based on ICA Algorithm

#### 4.2.1. ICA

ICA was proposed to solve the problem of blind source separation [20] (BSS). It has developed into a multidimensional signal processing technology. In terms of image feature extraction, it is an extension of PCA, focusing on image The high-order statistical characteristics make the components of the transformed image independent of each other and make more effective use of the essential characteristics of the image.

The research of ICA algorithm originates from blind source separation, which is a process of recovering independent source signals from the source signal only from the observation signal according to the statistical characteristics of the input source signal when the source signal and the transmission channel parameters are unknown. When the ICA algorithm is applied to image feature extraction, it realizes the separation of images and generates a set of independent source images, and uses these source images as a set of base images of the image set, that is, the images in the image set can be composed of these independent base images. The linear superposition of the image under different combination coefficients minimizes the redundancy of the image pixel gray value and extracts the essential characteristics of the image.

The article "Research on Image Feature Extraction Algorithm of the Egg and Egg White Protein Thermal Gelation Based on PCA/ICA" was published in 2022. Journal: Comput Intell Neurosci.

Let *s*=[*s*_1_, *s*_2_,…*s*_*m*_]^*T*^ be *m* unknown independent source signals with zero-mean value, and *X*=[*x*_1_, *x*_2_,…*x*_*n*_]^*T*^ are *n* random observation signals formed by linear mixing of source signals. Then there are

(11) $$\begin{array}{c} X=\text{AS}. \end{array}$$

And is

(12) $$\begin{array}{c} x_{i}=\sum_{j=1}^{m}a_{ij}s_{j}. \end{array}$$

Among them, *i*=1,2,…, *n*, *j*=1,2,…, *m*, *A*=[*a*_1_, *a*_2_,…, *a*_*n*_] is a full-rank matrix of size *n*×*m*.

Let *Y*=[*y*_1_, *y*_2_,…, *y*_*m*_] be the estimated signal, then

(13) $$\begin{array}{c} Y=\text{WS}\\ =\text{WAS}. \end{array}$$

Among them, W is called the unmixing matrix. When WA is the identity matrix, the estimated signal is an independent source signal, and because the non-Gaussian nature of random variables is closely related to statistical independence. According to the central limit theorem, when a group of random variables with the same mean and variance act together, the result will be close to the Gaussian distribution, that is, the non-Gaussian of the source signal is stronger than that of the observation signal. Therefore, when the non-Gaussian is maximized, the estimated signal is closer to the source signal. The ICA algorithm uses the unmixing matrix corresponding to the strongest non-Gaussian as the projection direction that ICA seeks based on the high-order statistical characteristics of *X* to estimate the independent source signal S and realize the separation of the independent sources.  Figure 7 is a simple diagram of the ICA model.  Figure 8 is an example of ICA used for blind source separation.  Figure 7(a) uses four basic signals such as sinusoidal signals as independent source signals.  Figure 7(b) is the result of linearly mixing the source signal as the observation signal.  Figure 7(c) is the estimated signal separated by ICA. It can be seen from Figure 8 that the ICA algorithm can be effectively used for blind source separation.

The ICA algorithm is different from the PCA algorithm, which regards the signal as a Gaussian distribution and only focuses on the second-order statistics of the signal, but focuses on the high-order statistics of the signal to study the independent relationship between the signals, so the ICA algorithm is more in line with the essential characteristics of image data. Since Hyvarinen et al. published a milestone paper in 1995 and proposed the Fast ICA algorithm, the algorithm has received extensive attention and has been applied to brain signals, speech signals, target detection, image processing, and other fields.

The two-dimensional image is vectorized to form an image signal. It can be considered that the image signal is formed by a set of linear aliasing of statistically independent base images. The base images are separated by the Fast ICA algorithm to form a feature subspace. Each image is in the feature subspace. Projection in the space achieves the purpose of extracting image features.

The article "Research on Image Feature Extraction Algorithm of the Egg and Egg White Protein Thermal Gelation Based on PCA/ICA" was published in 2022. Journal: Comput Intell Neurosci.

The feature selection after the independent component feature extraction is an important factor in determining the subsequent classification and recognition of the image. How to use fewer features to quickly obtain a higher classification and recognition rate is a key issue to test the feature extraction algorithm. In the actual feature extraction of images, it is required that the extracted features have as large a difference as possible for images that do not belong to the same category and as small as possible for images that belong to the same category. Since the signals separated by Fast ICA are disordered, the intra-class distance function is introduced to optimize the features.

Assuming that the image set has *M* types of images, and each type of image is composed of N images, *U*_*j*_ is called the mean value of the distance within the *j*th feature of the *M* type, which can be expressed as follows:

(14) $$\begin{array}{c} U_{j}=\frac{1}{\text{MN}\left(N-1\right)}\sum_{i=1}^{M}\sum_{u=1}^{N}\sum_{\begin{array}{c} v=1\\ v\neq u \end{array}}^{N}\left|a_{\left(i-1\right)N+u,j}-a_{\left(i-1\right)N+v,j}\right|. \end{array}$$

Among them, *a*_*i*,*j*_ is the *j* features of the *i*th image. In the same way, the mean value *V*_*j*_ of the distance between classes of the *j*th feature *M* class can be expressed as follows:

(15) $$\begin{array}{c} U_{j}=\frac{1}{\text{MN}\left(N-1\right)}\sum_{p=1}^{M}\sum_{\begin{array}{c} q=1\\ q\neq p \end{array}}^{N}\left|\frac{1}{N}a_{\left(p-1\right)N+u,j}-\frac{1}{N}a_{\left(q-1\right)N+v,j}\right|. \end{array}$$

The evaluation factor *β*_*j*_ of the *j*th feature is expressed as follows:

(16) $$\begin{array}{c} \beta_{j}=\frac{U_{j}}{V_{j}}. \end{array}$$

The value of *β*_*j*_ reflects the accuracy of the *j*th feature for classification. When *β*_*j*_ is small, it means that the distance between classes is greater than the distance within the class, which makes it easier to distinguish different classes. On the contrary, when *β*_*j*_ is large, it means that the distance between classes is larger. The distance is greater than the distance between classes, and it is not easy to classify. Therefore, the evaluation factors of all features can be sorted, and some features with fewer evaluation factors that are most conducive to target classification are selected as the most characteristic set for the final classification.

The article "Research on Image Feature Extraction Algorithm of the Egg and Egg White Protein Thermal Gelation Based on PCA/ICA" was published in 2022. Journal: Comput Intell Neurosci.

#### 4.2.2. Subpattern-ICA

The Subpattern-ICA algorithm is based on the ICA algorithm with the selection of the objective function, image preprocessing, and feature optimization. First, the training set image is divided into blocks, as shown in Figure 9, the image is equally divided into multiple sub-blocks without overlapping, and then the corresponding sub-blocks are vectorized to form the training set sub-model. Usually, the local change trend in the image is not the same, so the classification contribution of each training set sub-model to the entire training set is not the same, and due to factors such as occlusion, expression, lighting, the reliability of the classification of each training set sub-model is also inconsistent. So Subpattern-ICA introduces the concept of adaptive weights. After using PCA independently for each training set sub-model, each training set sub-model is classified and recognized, and the classification recognition rate is obtained and normalized as the weighted value of the classification rate of each submodel in the final classification voting stage.  Figure 10 is a visualization of the three images in the egg white protein image database and the median image and average image in the database as the test images to calculate the weights of each sub-model. The lighter the color in the figure, the greater the weight, and the greater contribution to the overall classification rate.

The main steps of the Subpattern-ICA algorithm are as follows:

**Step 1 .**

The training image set is divided into N sub-blocks, and the corresponding sub-blocks form a sub-model;

**Step 2 .**

Use the Fast ICA algorithm to obtain the characteristic projection matrix for each sub-block model;

**Step 3 .**

Project the image in the sub-model with the corresponding feature projection matrix to extract features;

**Step 4 .**

Divide the test image set image into N sub-blocks according to Step 1. Each sub-block image uses the feature projection matrix of the corresponding training sub-model in step 2 to extract features, and uses the nearest neighbor method to compare the test images based on the sub-model image features The set of sub-block images are classified, and the normalized sum of the votes of each sub-model is used to determine which category the test image set images belong to.

The Subpattern-ICA algorithm uses the idea of sub-patterns to limit the impact of each sub-block image on the overall image within the sub-block image, so that even if the image has serious lighting, expression, and occlusion changes, the changes are reflected in the sub-block image. It will not interfere too much in the feature extraction and classification of the image as a whole. This improves the algorithm's robustness to local changes and improves the algorithm's feature extraction effect.

The article "Research on Image Feature Extraction Algorithm of the Egg and Egg White Protein Thermal Gelation Based on PCA/ICA" was published in 2022. Journal: Comput Intell Neurosci.

## 5. Results

### 5.1. Simulation Experiment and Result Analysis

The hardware configuration of the PC used in this article is as follows: the CPU model is Intel's Core IS 6600K, the main frequency is 3.SGHz, and the memory is 16 GB DDR4; the software environment is as follows: MATLAB version 2021a; the algorithm is tested on the egg white gel image database. The experiment is used to compare the performance of feature extraction between PCA and Wavelet PCA algorithms, as well as ICA and Subpattern-ICA. In the experiment, three random division methods were selected for the image set of the egg white gel database to verify the feasibility of the algorithm. In the experiment, the nearest neighbor method was used as the classifier, and all the experimental results were averaged after being executed ten times.

### 5.2. Simulation Experiment and Result Analysis

The egg white protein image database is obtained by crawler extraction based on the characteristics of the image through big data, including rich images of a variety of egg white proteins in different states, totaling 10,000 images. The gray level of the original egg white is 256, with a total of 320×243 pixels. In this experiment, all the images are first cropped to a size of 128×128.

Figure 11 shows 10 images of the egg white state in the egg white protein image database. In this experiment, the egg white protein image database is used as the input image set, and P images in different states of the egg white are randomly selected to form the training image set, and the remaining images are used as the test image set images. The values of P are 1, 4, and 5, that is 1 train, 4 train, and 5 train.

It can be seen from Table 1 that the recognition rate of all algorithms will increase as the number of training increases. Overall, the recognition rate of Wavelet PCA is higher than that of PCA, while the recognition rate of 2DPCA is higher than that of Wavelet PCA and PCA. This is because Wavelet PCA first uses wavelet transform to extract the detailed information of the image, while PCA only uses the gray information of the image. In addition, 2DPCA uses the image matrix as a whole for covariance calculation, taking into account the structural information of the image, which is more effective. It is more representative of the image, and the recognition rate is higher. It can be seen from Figure 12 that the egg white protein image database has changes under the influence of light, and 2DPCA is more effective in such high-change images. Since 2DPCA is different from the other two algorithms in calculating the feature dimension, Figure 12 here shows the curve of the recognition rate of Wavelet PCA and PCA with the feature dimension in the two cases of 1 train and 5 train.

The article "Research on Image Feature Extraction Algorithm of the Egg and Egg White Protein Thermal Gelation Based on PCA/ICA" was published in 2022. Journal: Comput Intell Neurosci.

It can be seen from the figure that in Strain, the two algorithms are relatively stable and remain unchanged after reaching a higher recognition rate. It can be seen that Wavelet PCA maintains a leading position compared with PCA. In the 1 train with a small number of samples, Wavelet PCA is also better than PCA.

In this experiment, the egg state image database is the egg white protein image database, and the sub-databases with characteristic types and obvious characteristics are used as the input image set. P images of each egg white in the solidification state at different temperatures are randomly selected to form the training image set. The remaining images are used as test images and the value of P is S, which is recorded as Strain.  Figure 13 shows the variation curve of the recognition rate of ICA and Subpattern-ICA with the feature dimension under 5 train. It can be seen from the figure that in the 5 train, both algorithms can achieve a higher recognition rate in a smaller feature dimension, and remain unchanged, with good robustness. However, it can be clearly seen from the figure that when the number of dimensions is small, the recognition rate of Subpattern-ICA stays ahead of ICA and can reach stability faster.

Table 2 shows the classification and recognition results of ICA and Subpattern-ICA in Strain. It can be seen from the table that the recognition rate of these two algorithms will increase with the increase of the feature dimension. On the whole, the recognition rate of Subpattern-ICA is higher than that of ICA. This is because Subpattern-ICA first divides the first image into blocks, and each sub-block uses ICA for feature extraction. It takes into account the structural information of the image but is not sensitive to local changes and can better represent the image, so the recognition rate is higher.

Consistent with the experimental results of the egg state image database in Experiment 1, it can be seen from Table 3 that the recognition rate of these two algorithms will increase with the increase of the feature dimension. On the whole, the Subpattern-ICA algorithm can better represent the image, the recognition rate is higher than that of the ICA algorithm, and it can quickly reach stability, and has good robustness.

It can be seen from the above two experimental results that the above two algorithms can be used for image feature extraction, and the recognition rate of the Subpattern-ICA algorithm and the image feature extraction proposed in this section are better.

The article "Research on Image Feature Extraction Algorithm of the Egg and Egg White Protein Thermal Gelation Based on PCA/ICA" was published in 2022. Journal: Comput Intell Neurosci.

The PCA-based image feature extraction algorithm is a classic image feature extraction algorithm. After the image matrix is vectorized, the covariance matrix is eigenvalue decomposed, and the eigenvector is used as the feature projection matrix. The algorithm is simple and easy to implement, and has been widely used in various fields. Usually, the image is a two-dimensional matrix, and the dimensionality of the image will be very high after vectorization. The direct use of feature extraction makes the algorithm too complex, resulting in unsatisfactory image extraction. On this basis, before using PCA for feature extraction, Wavelet PCA first performs wavelet transformation on the image to extract wavelet coefficients, which greatly reduces the data dimension used for PCA. This algorithm has good feature extraction effect for images with low changes.

The image feature extraction algorithm based on ICA realizes the separation of images, generates a set of independent source images, and uses these source images as a set of base images in the image space to perform feature extraction on the images. The algorithm considers the high-order statistics of the image, which is more in line with the non-Gaussian nature of the image. But the disadvantage is that the algorithm still needs image vectorization processing, ignoring the internal structure information of the image, and the iterative speed is too slow when the algorithm constructs the objective function and optimizes the objective function, which affects the real-time performance of the algorithm. Based on this, Subpattern-ICA is proposed, which uses the idea of sub-patterns to divide the image into sub-patterns, and then uses ICA for feature extraction for each sub-pattern independently, and finally uses adaptive-weighted voting to determine the classification of the image. The algorithm uses the structural information of the image, improves the robustness of the algorithm for local changes, and improves the feature extraction effect.

## 6. Conclusion

This article tries to find the optimal parameter combination through traditional parameter adjustment, studies the physical and chemical changes in the egg white, and obtains the optimal parameters through different image state characteristics during the change. This article focuses on the thermal gelation of the egg white protein. In the image feature extraction algorithm, through the analysis of the simulation experiment results, Wavelet PCA is obtained by extracting wavelet coefficients, which greatly reduces the data dimensionality used for PCA, has a good feature extraction effect for images with low changes, and improves the complexity of the PCA algorithm. The improved PCA algorithm is too high, resulting in unsatisfactory image feature extraction. The improved algorithm Subpattern-ICA uses the idea of sub-patterns to divide the image into sub-patterns, uses the structural information of the image, improves the robustness of the algorithm for local changes, and improves the feature extraction effect. Through this research, it can be seen that PCA and ICA have enhanced the distinguishing ability of features to varying degrees, which can enrich the connotation of image feature extraction and solve the problem of image extraction in different states. In addition, the number of image data extracted by the algorithm used in this article is complicated. When the algorithm is simulated and verified, there will inevitably be shortcomings. In the future, similar research should establish an infrared database for feature extraction and classification in the laboratory to verify the feasibility of the algorithm.

The article "Research on Image Feature Extraction Algorithm of the Egg and Egg White Protein Thermal Gelation Based on PCA/ICA" was published in 2022. Journal: Comput Intell Neurosci.

## Figures and Tables

**Figure 1:** The influence of gel temperature on the gel strength of the egg white.

**Figure 2:** The effect of gel time on the gel strength of the egg white.

**Figure 3:** Schematic diagram of principal components of two-dimensional random data.

**Figure 4:** Schematic diagram of image matrix vectorization.

**Figure 5:** Example of the egg and egg white protein.

**Figure 6:** Image wavelet decomposition.

**Figure 7:** Schematic diagram of ICA model.

**Figure 8:** An example of ICA used for blind source separation.

**Figure 9:** Block diagram.

**Figure 10:** Schematic diagram of adaptive weights.

**Figure 11:** Ten image state samples of egg whites in the egg white protein image database.

**Figure 12:** The recognition result of the algorithm in the egg white protein image database. (a) 1 train (b) 5 train.

**Figure 13:** The recognition result in the image database of the egg state of the algorithm.

**Table 1:** In the egg white protein image database, the highest recognition rate obtained after each algorithm is stabilized (%).

Egg white protein image database	1 train	4 train	5 train
PCA	43.07	62.00	63.89
Wavelet PCA	45.47	62.57	62.55

**Table 2:** In the egg state image database, the recognition rate corresponds to the feature dimension (%).

Egg state image database	10	20	30	40	50	60	70	80	90	100
ICA	55.5	69.65	76.95	81.05	83.45	85.15	85.95	87.15	87.75	88.8
Subpattern-ICA	85.6	87.55	88.35	89.3	89.65	89.65	89.75	89.65	89.75	89.45

**Table 3:** In the egg white protein image database, the recognition rate corresponds to the feature dimension (%).

Egg white protein image database	10	20	30	40	50	60	70	80	90
ICA	60.13	64.4	65.13	65.07	64.8	64.53	65.33	66.67	66.53
Subpattern-ICA	64.8	66.53	66.8	67.07	67.2	67.2	67.2	67.2	67.2

The article "Research on Image Feature Extraction Algorithm of the Egg and Egg White Protein Thermal Gelation Based on PCA/ICA" was published in 2022. Journal: Comput Intell Neurosci.

## Data Availability

The dataset can be accessed upon request.

## References

[1] Carreira-Perpinan M. A. (1997). A review of dimension reduction techniques.

[2] Jolliffe I. T. (2002). *Principal Component Analysis*.

[3] Shlens J. (2009). *A Tutorial on Principal Component Analysis*.

[4] Hyvärinen A., Oja E. (2000). Independent component analysis: algorithms and applications. *Neural Networks*.

[5] He X. F., Niyogi P. (2003). Locality preserving projections. *Neural Information Processing Systems*.

[6] Etemad K., Chellappa R. (1998). Discriminant analysis for recognition of human face images. *Journal of the Optical Society of America. A*.

[7] Martinez A. M., Kak A. C. (2001). PCA versus LDA. *IEEE Transactions on Pattern Analysis and Machine Intelligence*.

[8] Zhang D., Frangi A. F. (2004). Two-dimensional pca: a new approach to appearance-based face representation and recognition. *IEEE Transactions on Pattern Analysis and Machine Intelligence*.

[9] Nagabhushan P., Guru D. S., Shekar B. H. (2006). Visual learning and recognition of 3D objects using two-dimensional principal component analysis: a robust and an efficient approach. *Pattern Recognition*.

[10] Zuo W., Zhang D., Wang K. (2006). An assembled matrix distance metric for 2DPCA-based image recognition. *Pattern Recognition Letters*.

[11] Xang L. (2006). On image matrix based feature extraction algorithms. *IEEE Transactions on Systems, Man and Cybernetics, Part B (Cybernetics)*.

[12] Haiping Lu H. P., Plataniotis K. N., Venetsanopoulos A. N. (2008). MPCA: m principal component analysis of tensor objects. *IEEE Transactions on Neural Networks*.

[13] Wang H., Ahuja N. (2008). A tensor approximation approach to dimensionality reduction. *International Journal of Computer Vision*.

[14] Chen C. M., Zhang S. Q., Chen Y. F. Face recognition based on MPCA.

[15] Wu G., Zhang P., Wang R. (2008). Independent component analysis and its application status in image processing. *Computer Engineering and Applications*.

[16] Han J., Chi K., Yeon Y. (2005). Aquaculture feature extraction from satellite image using independent component analysis. *Machine Learning and Data Mining in Pattern Recognition*.

[17] Huang Q. H., Wang S., Liu Z. (2007). Improved algorithm of image feature extraction based on independent component analysis. *Electronic Engineering*.

[18] Gan J. Y., Li C. Z. (2007). Face recognition based on wavelet Transform,Two-dimensional principal component analysis and independent component analysis. *Pattern Recognition and Artificial Intelligence*.

The article "Research on Image Feature Extraction Algorithm of the Egg and Egg White Protein Thermal Gelation Based on PCA/ICA" was published in 2022. Journal: Comput Intell Neurosci.

[19] Jiao Q. Face recognition method based on wavelet and PCA.

[20] Jiao X. (1996). General approach to blind source separation. *IEEE Transactions on Signal Processing*.

